# Identification and Classification of Prostate Cancer Identification and Classification Based on Improved Convolution Neural Network

**DOI:** 10.1155/2022/9112587

**Published:** 2022-07-18

**Authors:** Shobha Tyagi, Neha Tyagi, Amarendranath Choudhury, Gauri Gupta, Musaddak Maher Abdul Zahra, Saima Ahmed Rahin

**Affiliations:** ^1^Computer Science & Engineering, Manav Rachna International Institute of Research and Studies, Faridabad, 121001 Haryana, India; ^2^Department of IT, G.L Bajaj Institute of Technology & Management, Greater Noida, India; ^3^Department of Zoology, Patharkandi College, 788724, Karimganj, Assam, India; ^4^Department of Biomedical Engineering, SGSITS, Indore, India; ^5^United International University, Dhaka, Bangladesh; ^6^Computer Techniques Engineering Department, Al-Mustaqbal University College, Hillah, 51001, Iraq

## Abstract

Prostate cancer is one of the most common cancers in men worldwide, second only to lung cancer. The most common method used in diagnosing prostate cancer is the microscopic observation of stained biopsies by a pathologist and the Gleason score of the tissue microarray images. However, scoring prostate cancer tissue microarrays by pathologists using Gleason mode under many tissue microarray images is time-consuming, susceptible to subjective factors between different observers, and has low reproducibility. We have used the two most common technologies, deep learning, and computer vision, in this research, as the development of deep learning and computer vision has made pathology computer-aided diagnosis systems more objective and repeatable. Furthermore, the U-Net network, which is used in our study, is the most extensively used network in medical image segmentation. Unlike the classifiers used in previous studies, a region segmentation model based on an improved U-Net network is proposed in our research, which fuses deep and shallow layers through densely connected blocks. At the same time, the features of each scale are supervised. As an outcome of the research, the network parameters can be reduced, the computational efficiency can be improved, and the method's effectiveness is verified on a fully annotated dataset.

## 1. Introduction

Most common among male cases in the latest global cancer statistics is lung cancer (14.5%), followed by prostate cancer (13.5%), the incidence of cancer in men, with the highest disease which is prostate cancer in more than 100 countries [1]. In the biography during the traditional diagnosis of prostate cancer, pathologists using needle biopsy to obtain case samples were obtained, pathological images were obtained after H&E staining, and microscopy was performed. To observe the tissue morphological pattern of the cells, it is necessary to confirm whether there is cancer in the tissue exists and is Gleason rated [2].

The Gleason grading model is a widely accepted and recognized standard in the evaluation of prostate cancer tissue microarrays [3]. It has been developed since 1966 and has been revised many times by the International Society of Urology and has been used in clinical practice. This stage is not only a pathological evaluation index, but also provides a reliable basis for doctors to diagnose in clinical diagnosis [4]. Sections containing biopsies can show the morphological organization of the glandular structures of the prostate. In low-grade tumors, the epithelial cells remain glandular structures, whereas in high-grade tumors, glandular structures are eventually lost. Prostate cancer's microarray tissue is divided into 5 growth patterns, 1 to 5, corresponding to different cell tissue morphology with better prognosis. Basically, there is no difference between normal tissue and poor prognosis. According to the proportion of the growth pattern, the growth pattern of a pathological section is divided into primary structure and secondary structure. The final score is obtained by adding the primary structure and secondary structure and classified into different prognosis groups according to the different scores, when not more than 6 points usually have better prognostic results. As shown in Table 1, five different prognostic groups were classified in the latest modified Gleason grading model: G1 when the score is not higher than 3 + 3; G2 for 3 + 4; G3 for 4 + 3; G4 for 3 + 5, 5 + 3, and 4 + 4; and G5 for higher scores. As shown in Figure 1, they represent benign Gleason scores of 6, 8, and 10, respectively.

The commonly used method in the Gleason automatic grading system for prostate cancer is to extract the feature organization and then classify the selected features using such as SVM (support vector machine), random forest, or Bayesian classifier. In these three methods, SVM is a supervised machine learning algorithm, whereas Bayesian classifier is an analytical paradigm that describes probability values as logics based on conditions conditional logic rather than long-run frequency range, and random forest is a supervised learning classification method and regression that randomly uses subsets of data and is inherently suitable for multiclass concerns. All of them can be employed in the classification of features in general. Reference uses ResNet18 as the basic model and believes that neural networks can be divided into distinguishing networks and generating networks [4].

The discriminative network adopts a classification model. This study first uses the texture features of glands to identify the presence of individual glandular structures; then, the texture features and morphometric obtained from glandular units are applied to the classification stage, and finally the images are labeled as grades 1 to 5 [5]. The literature shows that the texture features of the image are represented according to the different power spectra of the image [6].

Classifiers assign different Gleason scores. In addition to this, another method is based on deep learning, especially convolutional neural networks (convolutional neural networks), and neural network (CNN), which can perform both feature learning and classification steps in one framework and achieve better results when the training data reaches a certain size, without being overly dependent on manual annotation [7]. The development of deep learning and computer vision has made CAD (computer auxiliary diagnostic systems) that are used in medical clinical treatments [8, 9]. The study used inceptionv3 to train 120,000 images and reached the expert level of dermatologists through the classification algorithm [10]. This study used a deep network classifier to predict the probability of diagnosis and referral after training tens of thousands of scans on histograms with confirmed diagnosis and optimal referral [11]. Convolutional neural networks (CNN) notably uses both feature learning and classification processes in a single framework and produces better results when this technique is employed over images that are obtained using various scanning techniques like MRI and PET scans and thus helps in better prediction and diagnosis of prostate cancer. Compared with the fully convolutional neural network (FCN), U-Net has more advantages in medical image processing as it has its roots in the convolutional network. It was developed for the segmentation of biomedical images with its vast application in the segmentation of brain site prediction in protein binding, liver, and biomedical image reconstruction. Its design was improved and expanded so that it could operate with less trained images to provide a more detailed segmentation method. Both share a classic idea, encoding and decoding (encoder-decoder); U-Net Net's network architecture is completely symmetrical on both sides and uses concatenation, which is different from FCN in that FCN uses summation [12, 13]. Fully convolutional networks are a type of structure commonly employed for feature extraction, also known as classification problems. The only locally linked layers of FCN are used that constitutes of convolution, filtering and data augmentation. There are fewer variables because dense layers are not utilized that can make networks faster to train. Due to the fact that all connections are local, an FCN can manage a broad set of image dimensions for providing assistance in feature extraction.

Due to being easily affected by subjective factors among pathology expert observers, manual viewing is labor-intensive, time-consuming, and inefficient, and there are differences in the ratings of the same slice among different observers [14]. With the aging of the population, the number of prostate cancer patients is increasing year by year, and the number of people who need biopsy is also increasing; the observation range of CAD tools is all areas of the slice, and the advantage of CAD tools is to avoid missed inspections caused by manual observation; and CAD tools are only compatible with internal algorithms [15]. It has nothing to do with labor intensity and time and can reuse computer resources to provide reproducible results, which can greatly improve the efficiency of diagnosis and treatment and ease the tension between doctors and patients [16, 17].

Different from the classifier algorithm, this paper proposes a Gleason grading study of prostate cancer tissue microarray region segmentation based on convolutional neural network, as shown in Figure 2, which has great clinical significance in the diagnosis and treatment of prostate cancer. Many studies have shown that region segmentation can be successfully applied in clinical trials [18, 19]. Most studies only focus on the distinction between Gleason 3 and Gloason 4. The research scope of this paper covers all types of benign and Gleason 1~5, and the scope is wider [18]. The difference from the segmentation of MR images and X-ray images is that the segmentation of tissue microarray images is based on cell morphological tissue and the difficulty coefficient of identifying growth patterns between different cell tissue morphologies, especially Gleason grades 3 and 4, is high, in the presence of cancer, particularly prostate [19, 20]. Furthermore, X-ray images vary from histopathology in that histology images possess a high amount of items of interest like cell features, e.g., nuclei that are widely distributed and accompanied by tissue and organs. X-ray image processing, on either hand, focuses primarily on a few tissues in the image that are more reliable in their location. Histology pictures, on either hand, are typically taken at a much lower incredible characteristics; the histology magnification extent is sufficient to allow some assessment at the cell level, such as nucleus measuring and identifier of gross malformations in the nucleoplasm; the lower magnifying level enables evaluation at the tissue level; therefore, due to these features possessed in the images provided by the histology, medical field is much reliable in this technique for the detection and investigation of malfunctioned cells that may be cancerous for the further prevention of fatal diseases.

The proportion of cancerous tissue cells in the biopsy is not more than 1%, and the evaluation steps of the biopsy are cumbersome and error-prone, which will lead to the inability to give the correct Gleason rating in the process of prostate cancer detection [21, 22]. This research offers the YOLOv5x-CG real-time lesion diagnosis model to improve the lesion identification rate of colorectal cancer patients dealing with lung, breast, and prostate [23]. This research proposes an improved AlexNet-based image categorization model, with two specified block structures that are added to Alex-Net to extract specification of diseased images [24]. The novelty of this study is that a region segmentation model based on an improved U-Net network is proposed, which fuses deep and shallow layers through densely connected blocks. At the same time, the features of each scale are supervised. As an outcome of the research, the network parameters can be reduced, the computational efficiency can be improved, and the method's effectiveness is verified on a fully annotated dataset that is obtained for prostate cancer detection and investigation. However, this paper advances on the basis of the original U-Net improvements that were made to increase densely connected blocks, and after merging feature maps. The gradient path is added to make the calculation between the layers tend to be balanced, which not only improves the gradient of the original U-Net progress on the basis after the feature map is merged.

The network adds a gradient path so that the calculation between each layer tends to be balanced, which not only improves the gradient of the original U-Net network and the problem of low model feature utilization and prevents excessively repetitive information flow from occupying the memory flow. Training and testing are carried out on public datasets, and patients are diagnosed in Haikou People's Hospital. The verification is carried out on the existing prostate cancer pathological images of the Science Department, which makes the experimental results more realistic and reliable.

Organization: The paper is structured into several sections where the Introduction is the initial section followed by the second section which states the proposed methodology of the study. The 3rd module describes the experiment and result analysis followed by the last module conclusion.

## 2. Proposed Method

### 2.1. Data Preprocessing

The prostate tissue microarray images used in this study consist of two parts: The first part comes from a total of 886 public databases with detailed pathology expert annotations; the other part comes from the pathological sections of existing prostate cancer in the Department of Pathology, Haikou People's Hospital images, from which 135 were screened. These image data are divided into three groups: training group, validation group, and test group. The details of each group are shown in Table 2.

In histopathology, scanned samples usually have megapixels, and the current memory and video memory limit the training of the entire image, as shown in Figure 3; the original image size is 3,100 × 3,100 RGB images, to obtain the optimal experimental results; in this paper, for the obtained original prostate cancer tissue microarray images, firstly use the original grayscale processing of all image data used for testing, training, and verification, and then grayscale each original image. And the label map is divided into 100 nonoverlapping parts according to the corresponding order, and the size is 256 × 256.

### 2.2. Network Model

In the field of medical image segmentation, the commonly used network models are fully convolutional neural network (FCN), DenseNet, and U-Net. The U-Net network architecture can perform model training on the basis of insufficient datasets and can combine low-level information with high-level information. The original U-Net network model passes from the beginning to the end of the network stage in an end-to-end mode. Feature map integrates to solve the deformability of the gradient. After 4 times of down sampling, a total of 16 times, the corresponding up sampling is performed 4 times, and the feature information obtained in the down sampling process is restored to the same size as the original image. The corresponding stage adopts skip links so that the feature map can integrate the underlying information, making the segmentation and prediction results more accurate.

In a segmentation network, it can be described as an encoding stage U followed by a decoding operation R. When the input image is x, the model can be represented by g(x), and the formula is as follows:

(1) $$\begin{array}{c} g\left(x\right)=R\left(U\left(x\right)\right). \end{array}$$

*U* means to reduce the dimension of the input image x and encode the image content and *R* to reconstruct the obtained feature information back to the pixel space. The goal of the network architecture is to first down sample the input image and then up sample and finally performs the regression operation in the U-Net architecture. The previous layer needs to pass the learned feature information to the next layer through the convolution operation, but the connection between each layer is sparse. To make full use of the feature information of each layer of the network, dense connections are used to transfer information between layers, and the last layer can obtain rich feature information to realize feature information reuse. Concatenation of dimensions makes the total number of parameters smaller than traditional structures.

In this paper, part of the dense link module and part of the transition layer are added to the U-Net architecture. As shown in Figure 4, the underlying feature map is passed through part of the dense link block, and the new feature map fuses the output of the previous layer as the input of the next module. After each dense connection block, two convolution and feature fusion operations will be performed. The improved network architecture is shown in Figure 5. To improve the performance of the network and avoid the problems of overfitting and regular parameter selection, a BN layer and a ReLu activation layer are added after the convolutional layer. The ReLu layer can alleviate the problem of gradient disappearance and can train a deeper network than sigmoid, with high speed and low computational cost. Transformation and reconstruction can restore the influence of the normalization operation of this layer on the existing feature information. After introducing learnable reconstruction parameters, the BN layer is defined as follows:

(2) $$\begin{array}{c} \mu \text{B}=\frac{1}{m}\overset{\text{m}}{\underset{i=1}{\sum }}{\text{x}}_{\text{i}}, \end{array}$$

(3) $$\begin{array}{c} \sigma_{\text{B}}^{2}=\frac{1}{m}\overset{m}{\underset{i=1}{\sum }}{\left({\text{x}}_{\text{i}}-\mu_{\text{B}}\right)}^{2}, \end{array}$$

(4) $$\begin{array}{c} x_{i}=\frac{{\text{x}}_{\text{i}}-\mu_{\text{B}}}{\sqrt{\sigma_{B}^{2}}+\in }, \end{array}$$

(5) $$\begin{array}{c} y_{i}=\gamma x_{i}+\beta =BN_{\gamma ,\beta \left(x_{i}\right)}, \end{array}$$

where *μ* is the translation parameter, *σ* is the scaling function, *m* is the size of the block, and *γ* and *β* are the reconstruction parameters. The calculation results of the above formulas are the mean, standard deviation, normalization, and reconstruction transformation, respectively.

### 2.3. Loss Function

This paper optimizes the objective function by defining loss. The goal of the network architecture model design is to minimize the prime loss between the trained labels and the output layer of the network model. In the training process of this paper, sigmoid is used as the activation function of neurons, and each training label is independent. In the binary classification task, the binary cross entropy loss function is often used. The formula is as follows:

(6) $$\begin{array}{c} \text{BCE}=\frac{1}{n}\overset{n}{\underset{\text{i}}{\sum }}\left({\text{y}}_{\text{i}}\text{ In }{\text{y}}_{\text{i}}\right)+\left(1-{\text{y}}_{\text{i}}\right)\text{In }\left(1-{\ddot{\text{y}}}_{\text{i}}\right), \end{array}$$

Among them, *y*_i_ is the prediction result of the pixel point, and *y*_i_ is the real classification of the pixel point. Suppose that when the label is 1 and the prediction result is larger, the loss is smaller. In an ideal case, the prediction result is 1, and the returned loss is 0; otherwise, when the prediction result is 0, the smaller the prediction result, the smaller the loss. As shown in Figure 6, the prediction result has a good calculation effect when the data distribution is relatively balanced and has an adverse effect on the back propagation, which is easy to make the training unstable. In view of the obvious imbalance of pixel categories in this study, the use of binary cross-entropy loss function will be dominated by the class with more pixels. In previous experiments, when the loss function used binary cross-entropy as the loss function, the test set predicted the image results and not ideal.

The Dice function was originally proposed in V-Net [25]. It is more effective for the problem of unbalanced categories and is often used to calculate the similarity between two samples, with a value ranging from 0 to 1. Assuming that A and B represent the same set of pixels in the two contour regions, and then Dice is defined as follows:

(7) $$\begin{array}{c} Dice\left(A,B\right)=2\frac{\left|\text{A}\cap \text{B}\right|}{\left|\text{A}\right|+\left|\text{B}\right|}, \end{array}$$

It can also be expressed as

(8) $$\begin{array}{c} \text{Dice}=1-\frac{2\sum_{\text{i}}^{\text{n}}{\text{y}}_{\text{i}}{\ddot{\text{y}}}_{\text{i}}}{\sum_{\text{i}}^{\text{n}}{\text{y}}_{\text{i}}+\sum_{\text{i}}^{\text{n}}{\ddot{\text{y}}}_{\text{i}}}, \end{array}$$

When the target value and the predicted value are too small, the gradient will change drastically, which is not conducive to model training.

This paper combines the binary cross entropy loss function, and Dice BCE_ Dice_loss is used as the loss function of this experiment, and the formula is as follows:

(9) $$\begin{array}{c} L=\gamma Dice+\left(1-\gamma \right)BCE, \end{array}$$

## 3. Experiment and Result Analysis

### 3.1. Dataset

In this study, each trained object *x* must have a corresponding label *y*, and the label image with the same height and width as the input and output is selected to complete the semantic segmentation task. Semantic segmentation performed by convolutional neural networks is based on pixel level. Unlike classification algorithms, the output is a labeled image with a fixed value for each pixel. A total of 641 detailed annotated prostate cancer pathological slices were used for training the model, and 245 digital pathological slices were used for training, and a certain number were randomly selected in the validation set for evaluation. The test set was annotated by two pathology experts. Due to the large size of the original pathological slices, Matlab was used to grayscale each image, and then each image was divided into 100 nonoverlapping images of the same size. The image dataset after segmentation was expanded by 100 times. There are 88,600 pieces of data in the test set and the test set. Then, set the size to 256 × 256, rename each image from 0 codes in the order of position, and then send the preprocessed image data into the model. To better represent the performance of this study, several images were randomly selected from the validation cohort for prediction, and the results were compared with the ground truth.

### 3.2. Parameter Settings

In the training process of this paper, Adam optimizer is used for optimization, the learning rate (lr) is 0.001, and BCE_Dice_loss is selected as the objective function. On the test set, a mixture matrix and Cohen's Kappa metric are used.  Table 3 shows the parameter settings of each layer in the improved U-Net model.

### 3.3. Experiments and Results

This paper uses the Kappa coefficient to predict the results of the NU-Net model test consistency check with expert manual annotation results, the formula is as follows:

(10) $$\begin{array}{c} \text{Kappa}=1-\frac{\sum_{\text{i},\text{j}}{\text{w}}_{\text{i},\text{j}}{\text{O}}_{\text{i},\text{j}}}{\sum_{\text{i},\text{j}}{\text{w}}_{\text{i},\text{j}}{\text{E}}_{\text{i},\text{j}}}, \end{array}$$

(11) $$\begin{array}{c} w_{i,j}=\frac{{\left(\text{i}-\text{j}\right)}^{2}}{{\left(\text{M}-1\right)}^{2}}, \end{array}$$

Among them, M is the number of images. i and j represent different image categories: 1 ≤ I, j ≤ M, and Oi; j is classified as i by the first rater and classified as j by the second rater number. Ei refers to the expected number of images that the first rater is expected to label as class i and the second rater is expected to label images as class j.

To compare the performance of U-Net model with FCN and DenseNet before and after improvement, this paper trains and tests the above four models on the same training set and test set. FCN8 is based on a pretrained VGG16 model with a stride of 8; DenseNet is tested on the ImageNet dataset with a stride of 2; the U-Net model is based on a standard configuration; NU-Net adds a dense connection module.

In this study, 886 and 135 prostate cancer microarray tissue images were selected from the public dataset and the Radiology Department of Haikou People's Hospital, respectively, for preprocessing, with good pathologist annotations, which is divided into three parts: training set, test set, and validation set; the images in each dataset are independent and non-repeating. Through the pretrained FCN8 DenseNet, the original U-Net model, and the improved NU-Net model, 80 images randomly selected in the validation set are compared in the experiment, and the results are shown in Tables 4–7, and Figures 6–9.

Compared with the original U-Net model and the mainstream models in the other two segmentation algorithms, the improved NU-Net model shows good performance in different levels of Gleason pattern recognition, among which the original U-Net and DenseNet are in the recognition of the L averages of benign tissue and G3, G4, and G5 are 62.46% and 75.44%, respectively. The results show that the performance of the DenseNet model is better than that of U-Net on the dataset of this paper, and the worst performance is the FCN8 model. The L average value of the U-Net model with densely connected blocks has reached 78.71%, and the segmentation performance of Gleasons 3, 4, and 5 is improved to varying degrees compared with the original U-Net model.

To calculate the consistency between the experimental results of the improved NU-Net model and the ground truth of the manual viewing annotation results, this paper conducts experiments on the test set and uses the Kappa indicator for evaluation, and the model prediction results are consistent with the ground truth annotation results. The comparison between the model prediction and the ground truth is shown in Figure 9. The first row is the original image of the prostate cancer microarray tissue, the middle is the ground truth, and the last row is the prediction result of the improved NU-Net model in this study. From the perspective of sorting and segmentation effects, the segmentation results of NU-Net are roughly comparable to the ground truth. To better show the experimental results, label map according to different.

## 4. Conclusion

In this paper, an improved U-Net model is proposed to grade prostate cancer microarray tissue. The experimental results show that in the test set and the validation set, under the same evaluation reference standard, the experimental results of the model are in good agreement with the manual annotation results of pathologist's high similarity. In this paper, four different networks are tested on the validation set, and the results show that the improved NU-Net has the best segmentation effect in benign G3, GJJ4, and G5, with an L mean of 77.73%. The segmentation results of the NU-Net model on the test set are in good agreement with the pathologist's manual annotation results in different ratings such as benign, G1, and G2, with a Kappa value of 0.797. Previous research focused on the area divided into G3 and G4, Gleason's rating in this paper covers G1~G5, and the research is more comprehensive. The present study could be improved in several ways: First, it does not take into account for the most common pathologist errors in clinical diagnosis; the model focuses on prostate cancer microarray tissue grading, but other types of cell tissue may be present in biopsy results for a future perspective; and second, it does not account for the most common pathologist errors in clinical diagnosis experimental. The image data utilized in the dyeing is complete, with high definition and good image quality. Ideally, the system should be able to dye and process at the same time. External technological issues such as scanner calibration caused differences; each biopsy in this study was conducted separately by pathologists and deep learning models. Multiple biopsies are required in clinical practice in the future; also, the data used in the study were based on biopsies rather than patients, which could contribute to an overestimation of the new dimensions. From the patient's perspective, the learning model should be based on several needle biopsies and predict the Gleason grade.

## Figures and Tables

**Figure 1:** Gleason rating prognostic group distribution.

**Figure 2:** Gleason classification based on region segmentation.

**Figure 3:** Gray processing of microarray histopathological sections.

**Figure 4:** Densely connected blocks.

**Figure 5:** Improved network architecture.

**Figure 6:** Accuracy of Gleason segmentation results.

**Figure 7:** F1 score of Gleason segmentation results.

**Figure 8:** Precision of Gleason segmentation results.

**Figure 9:** Recall of Gleason segmentation results.

**Table 1:** Gleason rating prognostic group distribution.

Prognostic group	G1	G2	G3	G4	G5
				3 + 5	4 + 5
Score	<3 + 3	3 + 4	4 + 3	5 + 3	5 + 4
				4 + 4	5 + 5

**Table 2:** Distribution of Gleason scores in training, testing, and validation sets.

Test group	Total number of cases	Benign	G = 1	G = 2	G = 3	G = 4	G = 5
Test set	245	12	75	32	27	86	13
Training set	641	103	193	62	26	133	124
Validation set	135	3	42	31	24	14	21
Total	1021	118	310	125	77	233	158

**Table 3:** Parameter settings of each layer of the network model.

Parameter	Feature map size	Step size
Enter	256∗256	—
Densely connected blocks	256∗256	[3 × 3 Conv − 64] × 2
Max pooling layer	128∗128	2 × 2/2
Densely connected blocks	128∗128	[3 × 3 Conv − 128] × 2
Max pooling layer	64∗64	2 × 2/2
Densely connected blocks	64∗64	[3 × 3 Conv − 256] × 2
Max pooling layer	32∗32	2 × 2/2
Densely connected blocks	32∗32	[3 × 3 Conv − 512] × 2
Max pooling layer	16∗16	2 × 2/2
Densely connected blocks	16∗16	[3 × 3 Conv − 1024] × 2
Deconvolution layer	32∗32	2 × 2/2
Densely connected blocks	32∗32	[3 × 3 Conv − 512] × 2
Deconvolution layer	64∗64	2 × 2/2
Densely connected blocks	64∗64	[3 × 3 Conv − 256] × 2
Deconvolution layer	128∗128	2 × 2/2
Densely connected blocks	128∗128	[3 × 3 Conv − 128] × 2
Deconvolution layer	256∗256	2 × 2/2
Densely connected blocks	256∗256	[3 × 3 Conv − 64] × 2
Convolutional layer	256∗256	1 × 1 conv

**Table 4:** Comparison of accuracy of Gleason segmentation results of different models, %.

Model	Benign	G3	G4	G5
FCN8	**87.1**	**53.08**	**62.4**	**50.7**
DenseNet	**91.9**	**70.3**	**74.7**	**53.3**
U-Net	**95.1**	**48.5**	**75.4**	**55.6**
NU-Net	**96.3**	**83**	**82.3**	**56.2**

**Table 5:** Comparison of F1 score of Gleason segmentation results of different models %.

Model	Benign	G3	G4	G5
FCN8	87.19	53.13	62.46	50.75
DenseNet	91.99	70.37	74.77	53.35
U-Net	95.20	48.55	75.48	55.66
NU-Net	96.40	83.08	82.38	56.26

**Table 6:** Comparison of precision of Gleason segmentation results of different models %.

Model	Benign	G3	G4	G5
FCN8	68.01	41.44	48.72	39.59
DenseNet	71.75	54.89	58.32	41.62
U-Net	74.25	37.87	58.87	43.41
NU-Net	75.19	64.80	64.26	43.88

**Table 7:** Comparison of recall of Gleason segmentation results of different models %.

Model	Benign	G3	G4	G5
FCN8	68.35	41.65	48.96	39.78
DenseNet	72.11	55.16	58.62	41.82
U-Net	74.62	38.06	59.17	43.63
NU-Net	75.57	65.13	64.58	44.10

## Data Availability

The data shall be made available on request.
